RETRACTED

# Neural Network Optimal Routing Algorithm Based on Genetic Ant Colony in IPv6 Environment

**DOI:** 10.1155/2021/3115704

**Published:** 2021-07-13

**Authors:** Weichuan Ni, Zhiming Xu, Jiajun Zou, Zhiping Wan, Xiaolei Zhao

**Affiliations:** Guangzhou Xinhua University, Guangzhou, China

## Abstract

The traditional IPv6 routing algorithm has problems such as network congestion, excessive energy consumption of nodes, and shortening the life cycle of the network. In response to this phenomenon, we proposed a routing optimization algorithm based on genetic ant colony in IPv6 environment. The algorithm analyzes and studies the genetic algorithm and the ant colony algorithm systematically. We use neural network to build the initial model and combine the constraints of QoS routing. We effectively integrate the genetic algorithm and ant colony algorithm that maximize their respective advantages and apply them to the IPv6 network. At the same time, in order to avoid the accumulation of a lot of pheromones by the ant colony algorithm in the later stage of the network, we have introduced an anticongestion reward and punishment mechanism. By comparing the search path with the optimal path, rewards and punishments are based on whether the network path is smooth or not. Finally, it is judged whether the result meets the condition, and the optimal solution obtained is passed to the BP neural network for training; otherwise, iterative iterations are required until the optimal solution is satisfied. The experimental results show that the algorithm can effectively adapt to the IPv6 routing requirements and can effectively solve the user's needs for network service quality, network performance, and other aspects.

## 1. Introduction

With the rapid development of the Internet and the continuous increase in the number of network users, users' requirements for network service quality and network performance are also increasing. In the next generation of IPv6 networks, routing issues will become a hot issue in the field of network communication [1–4]. In the IPv6 network environment, users have higher requirements for network security, network quality of service (QoS), and so on. This requires routing algorithms running in the IPv6 protocol environment to have better security, reliability, and higher performance. The routing protocols used in IPv6 networks are mainly the routing protocol based on distance vector and the routing protocol based on link state [5, 6]. Both types of protocols need to periodically exchange information to maintain the correct routing table or network topology structure diagram of the network. However, the traditional IPv6 routing protocol is used in the resource-constrained IoT perception layer network. Switching a node from a dormant state to an active state will cause frequent changes in the topology, resulting in control information occupying a large number of wireless channel resources, increasing the energy consumption of the number of nodes, and shortening the life cycle of the network. At the same time, with the continuous increase in data traffic in the network, the intensity of router processing and calculation also increases accordingly, which will cause some node routers in the network to be in a high load state. Once the network traffic continues to increase, it will eventually cause network congestion, resulting in the router throwing a lot of packets, which reduces the service performance of the network and even causes the network to collapse.

RETRACTED

In view of the above problems, the next generation IPv6 network protocol has been analyzed and researched. We have systematically analyzed and researched the principles of the genetic algorithm and ant colony algorithm [7–10]. And based on it to improve and optimize, we use neural network to build the initial model and combine the constraints of QoS routing [11–14]. We propose a genetic ant colony routing optimization selection algorithm in the IPv6 environment. The routing algorithm not only can comprehensively use the constraints of QoS routing to solve the optimal route but also systematically analyze the genetic algorithm and the ant colony algorithm, effectively integrate and maximize their respective advantages, and select the best route in the IPv6 network. At the same time, in order to avoid that the ant colony algorithm accumulates a lot of pheromones in the later stage of the network, it tends to choose the side with more pheromone, and this paper introduces an anticongestion reward and punishment mechanism, which compares the search path with the optimal path. When the search time is too long and the search node exceeds the new threshold *λ*, it is regarded as the occurrence of node congestion. When the search path in the search algorithm is relatively smooth, we will reward it. And then, it is judged whether the result meets the condition, and the optimal solution obtained is passed to the BP neural network for training; otherwise, iterative iterations are required until the optimal solution is satisfied. Speed up the search speed of the algorithm while reducing unnecessary searches, so that the algorithm can still maintain a high optimization ability even in an environment where there is a “dead road” in the link.

## 2. Neural Network

We build a BP neural network to complete the classification task of cluster head nodes and common node features. BP neural network is a multilayer feedforward network trained by error propagation. The neural network consists of two parts: the forward transmission of information and the reverse transmission of errors [15–17]. A large number of neuron nodes are distributed in the neural network, and each neuron is connected by weights and thresholds to form a three-layer neural network structure. It includes an input layer, a hidden layer, and an output layer. BP neural network can approximate any nonlinear mapping relationship and has a good classification ability. It can well complete the classification based on the characteristics of wireless sensor nodes.  Figure 1 is a three-layer neural network model.

RETRACTED

The neural network adopts a nonlinear mapping parallel management mechanism, which has a high degree of self-learning ability, good generalization ability, and can quickly approximate any nonlinear mapping. However, the BP neural network also has certain shortcomings; that is, the BP neural network needs to train a large amount of sample data to determine the initial weight and threshold related parameters, which leads to the slow learning speed of the BP neural network and easy to fall into the local minimum. Therefore, this paper uses the BP neural network to initialize the system and determines the BP neural network topology through the wireless sensor network topology to obtain the initial population. Through the genetic ant colony algorithm, the optimal path is generated, a new population is generated, and it is judged whether the situation at this time requires repeated iteration. If the conditions are met, the obtained optimal solution is passed to the BP neural network for training; otherwise, iterations need to be repeated until the optimal solution is satisfied.

## 3. Analysis of Genetic Algorithm and Ant Colony Algorithm

Through the study of the two algorithms, it is found that in different stages, they have their own search advantages [18–20]. In the early stage of algorithm search, the genetic algorithm is obviously better than the ant colony algorithm. In the ant colony algorithm due to the lack of pheromone in the early stage, the search takes a lot of time to accumulate pheromone and choose the best path. The ant colony algorithm has been maintained at a relatively low search speed in the early stage. The ant colony algorithm has a positive feedback mechanism and a strong global convergence function in the later stage so that the algorithm has a good search efficiency in the later stage. The genetic algorithm has better global search capabilities, so its search speed is maintained at a relatively fast state in the early stage of the algorithm. However, in the later stage, the algorithm lacks a processing mechanism for the feedback information, resulting in a large number of unnecessary redundant iterations, which reduces the algorithm's search speed in the later stage.

RETRACTED

The following is the coordinate map of the city, and by observing the path selection of the genetic algorithm and the ant colony algorithm in the same environment, Figure 2 is the initial population corresponding to the city. Figures 3 and 4 are the optimal path diagram of the genetic algorithm and ant colony algorithm.

By observing Figures 5 and 6, we can see that the more iterations, the shorter the path length calculated by the system. And when the number of iterations reaches a certain amount, the optimal path of the two is basically unchanged. The evolutionary mechanism of the genetic algorithm is based on individual competition, and the search mechanism of the ant colony algorithm is a group cooperation under the pheromone conduction mechanism between ants. We can combine both to reduce the adjustment of parameters, avoiding a large number of blind iterations, generating populations in genetic algorithms, and speeding up the speed of the ant algorithm avoiding the exact solutions to the topical phase.

The algorithm first uses a genetic operator to perform a global fast search and then converts the obtained global search information into the initial value of the pheromone of the ant colony algorithm and uses the ant colony operator to complete the path selection.

## 4. The Proposed Algorithm

### 4.1. Genetic Operator: Global Fast Search

For an optimization problem, a certain number of candidate solutions (called individuals) can be abstractly represented as chromosomes so that the population can evolve to a better solution [21]. In each generation, the fitness of the entire population is evaluated, and multiple individuals are randomly selected from the current population (based on their fitness). We generate a new life population through natural selection and mutation, which will become the current population in the next iteration of the algorithm.

By observing Figures 7–9, we can see that there are countless “mountains” in the multidimensional surface, and these peaks correspond to local optimal solutions. And there will be a “mountain” with the highest altitude, so this is the global optimal solution. The task of the genetic algorithm is to climb to the highest peak as much as possible.

This article adopts the tree coding method; that is, the tree is composed of chromosomes from the source node to the destination node, and the genetic algorithm directly acts on the daily chromosomes.

RETRACTED

General QoS routing problems include multiple constraints, such as delay cost, bandwidth, delay jitter, and packet loss rate [22]. If you consider all factors when designing a specific routing algorithm, simplify it in combination with the actual situation. QoS routing mainly considers the three constraints of delay, bandwidth, and cost [23–25].

Time delay is as follows:

(1) $$\begin{array}{c} \text{Delay}\left(p\left(s,d\right)\right)=\underset{e\in p\left(s,d\right)}{\sum }D\left(e\right)+\underset{n\in p\left(s,d\right)}{\sum }D\left(n\right). \end{array}$$

*D*(*e*) : *E*⟶*R*^+^ delay on link *e*. *D*(*n*) : *V*⟶*R*^+^ delay on node *n*.

Bandwidth is as follows:

(2) $$\begin{array}{c} \text{Width}\left(p\left(s,d\right)\right)=\underset{e\in p\left(s,d\right)}{\min}\left\{B\left(e\right)\right\}. \end{array}$$

*B*(*e*) : *E*⟶*R*^+^ reservable bandwidth on link *e*.

Cost is as follows:

(3) $$\begin{array}{c} \text{Cost}\left(p\left(s,d\right)\right)=\underset{e\in p\left(s,d\right)}{\sum }C\left(e\right)+\underset{n\in p\left(s,d\right)}{\sum }C\left(n\right). \end{array}$$

*D*(*e*) : *E*⟶*R*^+^ cost on link *e*. *D*(*n*) : *V*⟶*R*^+^ cost on node *n*.

#### 4.1.1. Selection

This article adopts an elite retention strategy to establish an elite database [26]. The individuals in the elite pool are retained and passed on directly to the next generation to facilitate the selection of the next generation.

Delay constraints are as follows: Delay(*p*(*s*, *d*)) ≤ *D*_*p*_.

Bandwidth constraints are as follows: Width(*p*(*s*, *d*)) ≥ *W*_*p*_.

Cost: In the path that meets the above two conditions, Cost(*p*(*s*, *d*)) is the smallest.

Among them, *D*_*p*_ is the delay constraint and *W*_*p*_ is the bandwidth constraint.

According to the genetic mechanism of the elite retention strategy, this paper defines the fitness function formula as follows:

(4) $$\begin{array}{c} f=\frac{1}{\text{Cost}\left(p\left(s,d\right)\right)/\Phi \left[\text{Delay}\left(p\left(s,d\right)\right)-D_{p}\right]}. \end{array}$$

$\Phi \left(x=\right)\left\{\begin{array}{cc} 1 & x\leq 0\\ r & x>0 \end{array}\right.$, where Φ(*x*) is the penalty function, where the value of the penalty *r* determines the penalty *r* ∈ (0,1).

Inheritance is selected according to the size of *f*-value. The solution with large *f* fitness is more likely to be selected and inherited to the next generation, while the solution with small fitness will be eliminated from generation to generation. QoS routing meets the following constraints when selecting nodes.

#### 4.1.2. Crossover and Mutation

*Crossover Operator*. This article uses a single point crossover method. That is, two chromosomes select a common node as the crossover point and realize this function through the interchange of links, but if there are multiple common nodes, the first common node is selected to perform the crossover function.

RETRACTED

*Mutation Operator*. A node (except the source node and the destination node) is randomly selected from the chromosome as the mutation point, and the nodes after the mutation point are randomly selected from the nodes directly connected to it until the destination node. We use a normal distribution mutation. A normal distribution with a mean of zero and a predetermined standard deviation are used to generate random numbers, as shown in Figure 10:

### 4.2. The Best Time to Merge

End condition of the genetic algorithm is as follows: judge the best fusion time of the genetic algorithm and ant colony algorithm.

This paper defines the control function of the genetic algorithm: $C=1-\left(\left(\bar{\text{Cost}{\left[p\left(s,d\right)\right]}_{m}}\right)/\left(\bar{\text{Cost}{\left[p\left(s,d\right)\right]}_{m+1}}\right)\right)$. Among them, $\bar{\text{Cost}{\left[p\left(t,d\right)\right]}_{m}}$ is the average value of the group cost obtained after the *m*^th^ iteration of the genetic algorithm where 1 < *m* < the number of iterations of the genetic algorithm, by dynamically controlling the fusion timing of the genetic algorithm and the ant colony algorithm according to the change of the *C* value.

At this time, the solution obtained by the genetic algorithm is transformed into the initial value of the pheromone of the ant colony algorithm. *τ*^*S*^(*i*, *j*)=*τ*^*C*^(*i*, *j*)+*τ*^*G*^(*i*, *j*), where *τ*^*C*^(*i*, *j*) is a predetermined pheromone constant given by the environment. When the genetic algorithm is successfully transferred to the ant colony algorithm, the optimal solution set obtained by the genetic algorithm can be set through the formula: *τ*^*G*^(*i*, *j*)=(*k*/(cost[*p*(*s*, *d*)]*∗*cost[*p*(*i*, *j*)])). We use it to convert to pheromone. *k* is a constant, the path in the optimal set through the superposition of the pheromone of node *i* and node *j* is found, and finally a new *τ*^*G*^(*i*, *j*) is obtained.

### 4.3. Accurate Solution of Ant Colony Operator

According to the genetic algorithm, the premature stagnation of the ant colony algorithm is improved [27–29]. The initial value of the pheromone is set by the global search information *τ*^*G*^(*i*, *j*) obtained by the genetic algorithm, and the ant colony operator is started to solve the task scheduling accurately.

*Pheromone Initialization*. Pheromone formula is as follows: *τ*_*i*,*j*_=*τ*^*G*^(*i*, *j*)+*c*.

*τ* ^*G*^(*i*, *j*) is the pheromone concentration after genetic algorithm optimization, and *c* is the pheromone constant.

RETRACTED

First, a starting node is selected, all the ants are placed at the starting point, and all paths have the same pheromone content. Ant *k* selects the next mobile node according to the size of the pheromone distribution on each path. Then, *P*_*i*,*j*_^*k*^(*t*) is the probability of the *k*-th ant from node *i* to node *j* at time *t*, and its calculation formula is as follows:

(5) $$\begin{array}{c} P_{i,j}^{k}\left(t\right)\left\{\begin{array}{cc} \frac{{\left[\tau_{i,j}\left(t\right)\right]}^{\alpha }\cdot {\left[\eta_{i,k}\left(t\right)\right]}^{\beta }}{\sum_{r\subset \text{allowed}}{\left[\tau_{i,r}\left(t\right)\right]}^{\alpha }\cdot {\left[\eta_{i,r}\left(t\right)\right]}^{\beta }}, & j\in {\text{allowed}}_{k},\\ 0, & \text{otherwise.} \end{array}\right. \end{array}$$

*α* is the information heuristic factor, *β* is the hope heuristic factor, and allowed_*k*_ is the next selectable node. And it means that ant *k* moves from the current node to the next set of all possible nodes. According to the above content, *α* is a pheromone heuristic factor, which represents how much pheromone exists on the path. More pheromone means that there are more ants passing by the path, and vice versa. *β* is the expected heuristic factor, which represents the consideration of the importance of the ants in choosing the path node. The larger the value, the greater the probability of moving to this point. The heuristic function calculation method is as follows:

(6) $$\begin{array}{c} \eta_{i,r}\left(t\right)=\frac{1}{\text{Cost}\left(i,j\right)}. \end{array}$$

It can be seen from formula (6) that the heuristic functions *η*_*i*,*j*_(*t*) and Cost(*i*, *j*) are inversely proportional to each ant. The greater the cost of the link, the smaller the value of the heuristic function. When all the ants complete a cycle, the pheromone concentration on the link path needs to be updated by updating tab*u*_*k*_ to record the optimal solution set of the nodes currently traversed by ant *k*.

The first is the volatilization of pheromone, and the second is the release of pheromone by the ants on the side they pass. *ρ* is the pheromone volatilization coefficient, and 0 < *ρ* < 1, and the calculation formula is as follows:

(7) $$\begin{array}{c} \tau_{i,j}\left(t+n\right)=\left(1-\rho \right)\cdot \tau_{i,j}\left(t\right)+\rho \Delta \tau_{i,j}^{k}\left(t\right). \end{array}$$

Δ*τ*_*i*,*j*_^*k*^(*t*) is expressed as the concentration of the pheromone remaining on the path (*i*, *j*) by the *k*-th ant during the *t*-th iteration loop.

Here, ants are used to release pheromone every week after walking. Specifically, the pheromone is released after all ants have walked a circle so as to avoid the ants in the front from directly affecting the ants in the back.

RETRACTED

Pheromone release formula is as follows:

(8) $$\begin{array}{c} \Delta \tau_{i,j}^{k}\left(t\right)=\frac{Q}{\text{Cost}\left(p_{k}\left(s,d\right)\right)}. \end{array}$$

Q is a constant (set to 1) and Cost(*p*_*k*_(*s*, *d*)) is the total cost of selecting the link for the *k*th ant.

### 4.4. Congestion Avoidance Mechanism

In the later stage of the algorithm search, because the genetic algorithm has accumulated a lot of pheromones for the ant colony algorithm, the search path of the algorithm has been basically determined. And in the ant colony algorithm, the ant colony's choice of path tends to be the one with more pheromone, which leads to the accumulation of more ants on the optimal path. The original pheromone is too late to volatilize. At this time, new pheromone accumulates, which eventually exceeds the load capacity of the node, resulting in path congestion.

By introducing a new threshold *λ* in the search process, when searching for nodes, the search path is compared with the optimal path. When the search time is too long and the search node exceeds the new threshold *λ*, it is regarded as the occurrence of node congestion.

Mutation operations are performed on the ant colony, a normal distribution is set with node variance *σ* to perform mutation operations on some genes with a small probability, and the expression for generating new individuals is as follows:

(9) $$\begin{array}{c} \sigma \prime =\sigma eN\left(0,\Delta \sigma \right),\\ x\prime =x+N\left(0,\Delta \sigma \prime \right), \end{array}$$

where *x* is the next path node of the ant colony.

The fitness function is selected to calculate the fitness of the individual. In this paper, the minimum mean square error of the learning sample is selected as the fitness function. The formula is as follows:

(10) $$\begin{array}{c} f=\frac{1}{M}\overset{M}{\underset{i=1}{\sum }}\overset{q}{\underset{j=1}{\sum }}{\left(a_{ij}-e_{ij}\right)}^{2}. \end{array}$$

It judged whether it meets the requirements of the current optimal solution, and it is used as the next path node; otherwise, the path pheromone is updated. At this point, it shows that there is a more optimal solution. The pheromone release formula Δ*τ*_*i*,*j*_^*k*^(*t*) in the ant's node selection probability calculation formula is redefined, and the formula is as follows:

(11) $$\begin{array}{c} \Delta \tau_{i,j}^{k}\left(t\right)=\left\{\begin{array}{cc} \frac{Q}{\text{Cost}\left(p_{k}\left(s,d\right)\right)}, & \text{node smooth,}\\ -\;\mu *\left(\frac{Q}{n}\right), & \text{node congestion,}\\ 0, & \text{otherwise.} \end{array}\right. \end{array}$$

Values are assigned to the pheromone of its path according to different situations. *n* is the node of the search path, and *μ* is the reward and penalty coefficient of node congestion. When node congestion occurs in the search algorithm, it will be punished, so that other ants will reduce the use of the path, prompting the ants to select nodes that meet the QoS requirements near the path, thereby alleviating the load pressure of the path. When the search path in the search algorithm is relatively smooth, reward it, speed up the search speed of the algorithm, reduce unnecessary searches, and improve the search efficiency of the algorithm. At the same time, this allows the algorithm to maintain a high optimization capability even in an environment where there is a “dead road” in the link.

RETRACTED

### 4.5. Iteration Termination Condition

We pass the generated optimal solution to the BP neural network and judge whether the situation at this time requires repeated iterations. If the conditions are met, the optimal solution is passed to the BP neural network for training; otherwise, it needs to repeat iterations until the optimal solution is satisfied.

The output error *e*_*n*_ is determined by the predicted output *Y*_*n*_ and the actual output *O*_*n*_. The formula is as follows:

(12) $$\begin{array}{c} \;e_{n}=O_{n}-Y_{n}. \end{array}$$

The threshold and weight are updated according to the error *e*_*n*_.

(13) $$\begin{array}{c} \varpi_{ij}=\varpi_{ij}+\zeta H_{i}\left(1-H_{i}\right)X\left(i\right)\sum_{n=1}^{m}\varpi_{ij}e_{n}. \end{array}$$

Among them, *ϖ*_*ij*_ represents the weight between the *i*-th neuron in the input layer of the neural network and the *j*-th neuron in the hidden layer, *n* is the number of input nodes, *m* is the number of output nodes, and *H*_*i*_ is the value of the input layer of the neural network.

(14) $$\begin{array}{c} \varpi_{jk}=\varpi_{jk}+\zeta H_{j}e_{n}. \end{array}$$

Among them,  *ϖ*_*jk*_  represents the weight between *j* neurons in the hidden layer of the neural network and the *k*-th neuron in the output layer and *H*_*j*_  is the output of the hidden layer.

When the output error *e*_*n*_ obtained by the BP neural network processing reaches the preset ideal value, the algorithm is terminated.

## 5. Simulation

In order to test the effectiveness of the algorithm proposed in this article, this article uses MATLAB 2015b programming to simulate, the network topology structure adopts a random generation method, and the establishment of a network topology diagram that meets the constraints of QoS routing is shown in Figures 11 and 12. An initial population with a scale of 25 is generated; that is, an analog network with 25 network nodes is generated, where the four-tuple composed of the metrics of each node is delay cost, bandwidth, delay jitter, and packet loss rate. The four-tuple composed of the metric indicators of each link is delay cost, bandwidth, delay jitter, and packet loss rate. It is assumed that the source node is node 1 and the destination node is node 25.

RETRACTED

In order to verify the performance of the algorithm, we compare the delay data obtained by analyzing the article algorithm of the system with the literature algorithm [30] and the traditional algorithm and analyzing the performance of each algorithm. The data are the data of each algorithm measured under the same environment, and an average value is recorded every 100 times. The measured data are shown in Figure13.

By observing Figure 13, it can be seen that the delay time of the algorithm in this paper is the lowest at all time points and the overall delay time is maintained at about 0.2 s under the same environment, which has good stability. With the increase in time, the delay time of traditional algorithms is getting longer and longer. In the case of this low delay time, we record the energy balance in the system, and the data are shown in Figure 14.

By observing Figure 14, we can see that under different simulation time conditions, the node energy balance changes between the algorithm in this paper, the algorithm in the literature, and the traditional algorithm. The article algorithm adopts the anticongestion reward and punishment mechanism, and we can see that compared with the other two algorithms, it maintains a better selection mechanism at different time nodes and will not make the system use the node with the smaller remaining energy as the cluster head node to avoid the remaining energy imbalance between nodes.

By observing Figure 15, we can see that in the overall cost data of the system, the system cost using the article algorithm system is the lowest. And after the number of nodes reached 70, the system cost began to remain at a stable number, while traditional algorithms and literature algorithms still have an upward trend. Observing Figure 16, we can see that the convergence of the system using the article algorithm is maintained within a short period of time. As the number of nodes increases, the convergence time curves of the three algorithms all maintain an increasing trend but the convergence trend of the algorithm in this paper is the lowest.

## 6. Conclusion

In response to the existing IPv6 routing requirements, we propose a genetic ant colony routing optimization algorithm in the IPv6 environment. We use neural networks, and we effectively integrate the genetic algorithm and the ant colony algorithm through the constraints of the QoS network. This gives full play to their respective advantages. An anticongestion reward and punishment mechanism introduced by the algorithm can solve the network congestion problem while improving the search efficiency of the algorithm. Finally, the output error is used to judge whether the best effect is achieved, the iteration is ended, and the optimal solution is output. Experiments show that the algorithm can effectively prolong the network life cycle and avoid the imbalance of residual energy of system nodes. Compared with other traditional algorithms, this algorithm can well adapt to IPv6 routing requirements and can effectively call system resources.

RETRACTED

## Figures and Tables

**Figure 1:** Model of neural network.

**Figure 2:** Initial distribution map of the number of cities 50.

**Figure 3:** The search result of the genetic algorithm.

**Figure 4:** Iterative curve of the genetic algorithm.

**Figure 5:** The search result of the ant colony algorithm.

**Figure 6:** Iterative curve of the ant colony algorithm.

**Figure 7:** Curve optimal value.

**Figure 8:** Plane optimal value.

**Figure 9:** Three-dimensional optimal value.

**Figure 10:** Abrupt curve of normal distribution.

**Figure 11:** Network topology simulation model 1.

**Figure 12:** Network topology simulation model 2.

**Figure 13:** Data of each algorithm measured under the same environment.

**Figure 14:** Comparison of node energy balance of each algorithm.

**Figure 15:** The cost curve of the system.

**Figure 16:** The convergence time curve of the system.

## Data Availability

The data used to support the results of this study are obtained from the corresponding author upon request.
